The article "Differential regulation of wild-type and mutant alpha-synuclein binding to synaptic membranes by cytosolic factors" was retracted in 2021. Reasons: duplicated images; unreliable data.

# Differential regulation of wild-type and mutant alpha-synuclein binding to synaptic membranes by cytosolic factors

**DOI:** 10.1186/1471-2202-9-92

**Published:** 2008-09-22

**Authors:** Sabine Wislet-Gendebien, Naomi P Visanji, Shawn N Whitehead, Diana Marsilio, Weimin Hou, Daniel Figeys, Paul E Fraser, Steffany AL Bennett, Anurag Tandon

**Affiliations:** 1 Centre for Research in Neurodegenerative Diseases, University of Toronto, Toronto, Ontario, M5S 3H2 Canada; 2 Centre for Cellular and Molecular Neurobiology, University of Liege, 4000 Liege, Belgium; 3 Neural Regeneration Laboratory, Ottawa Institute of Systems Biology, Department of Biochemistry, Microbiology, and Immunology, University of Ottawa, Ottawa, K1H 8M5, Canada; 4 Institute for Biological Sciences, National Research Council of Canada, Ottawa, K1A 0R6, Canada

## Abstract

**Background:**

Alpha-Synuclein (α-syn), a 140 amino acid protein associated with presynaptic membranes in brain, is a major constituent of Lewy bodies in Parkinson's disease (PD). Three missense mutations (A30P, A53T and E46K) in the α-syn gene are associated with rare autosomal dominant forms of familial PD. However, the regulation of α-syn's cellular localization in neurons and the effects of the PD-linked mutations are poorly understood.

**Results:**

In the present study, we analysed the ability of cytosolic factors to regulate α-syn binding to synaptic membranes. We show that co-incubation with brain cytosol significantly increases the membrane binding of normal and PD-linked mutant α-syn. To characterize cytosolic factor(s) that modulate α-syn binding properties, we investigated the ability of proteins, lipids, ATP and calcium to modulate α-syn membrane interactions. We report that lipids and ATP are two of the principal cytosolic components that modulate Wt and A53T α-syn binding to the synaptic membrane. We further show that 1-O-hexadecyl-2-acetyl-*sn*-glycero-3-phosphocholine (C16:0 PAF) is one of the principal lipids found in complex with cytosolic proteins and is required to enhance α-syn interaction with synaptic membrane. In addition, the impaired membrane binding observed for A30P α-syn was significantly mitigated by the presence of protease-sensitive factors in brain cytosol.

**Conclusion:**

These findings suggest that endogenous brain cytosolic factors regulate Wt and mutant α-syn membrane binding, and could represent potential targets to influence α-syn solubility in brain.

## Background

The synuclein family of intrinsically unfolded proteins is composed of three homologous and evolutionarily-conserved members with poorly defined physiological roles [1]. Of these, α-synuclein (α-syn) has gained particular prominence due to its abundance in nerve terminals and its association with multiple neurodegenerative disorders including Parkinson disease (PD) [2]. α-Syn behaves as a peripherally associated membrane protein and can stably interact with synthetic phospholipid vesicles containing negatively charged head groups [3] via its amino-terminal domain, an amphipathic region comprising almost two-thirds of the protein and containing seven copies of an 11-residue repeat sequence [4]. Whereas the freely diffusible form of α-syn is natively unfolded, the N-terminal repeat region adopts an α-helical conformation upon binding to artificial vesicles and detergent micelles [3]. Numerous studies have revealed that the interaction of α-syn with phospholipid membranes, fatty acids, or detergent micelles alters the kinetics of its aggregation [4-9]. We and others have previously reported that synaptic α-syn *in vivo *is partitioned between both cytosolic and membrane-bound fraction [10-14]. However, despite the understanding of the conformational properties of membrane-bound α-syn, the biochemical mechanisms that mediate α-syn interaction with biological membranes are poorly understood, thereby limiting our understanding of α-syn's physiological role, as well as potential therapeutic approaches to moderate its misfolding and aggregation in disease.

In this study, we developed an *in vitro *assay to characterise the factor(s) involved in α-syn's binding to synaptic membranes (Figure 1A). Using this assay, we analysed the effects of cytosolic proteins, lipids, ATP and calcium on the modulation of α-syn membrane association. Our results revealed that ATP and lipids are two of the principal cytosolic components that modulate the α-syn binding to synaptic membranes. In addition, we report here that the binding of A30P α-syn to synaptic membranes improves significantly in the presence of endogenous cytosolic protein(s) and that the lower recovery of membrane bound A30P is likely due to a more transient interaction which can be stabilised by artificial cross-linking.

**Figure 1:** **(A) α-syn binding assay**. **Step 1**. Synaptosomes are prepared from α-syn^-/- ^mice and α-syn (human Wt and PD-linked A30P and A53T forms) is expressed and purified from E. coli. **Step 2**. Synaptic membranes (α-syn acceptor fraction) are prepared from intact synaptosomes using hypotonic buffer and incubated with purified α-syn (donor fraction) in presence or absence of α-syn^-/- ^(KO) cytosol. **Step 3**. Membrane and cytosol fractions are separated by centrifugation and the membrane proteins are analysed by western blotting. **(B) **Using the binding assay, KO synaptic membranes were incubated, for 10 min at 37°C, with 3 μg of Wt, A30P or A53T purified α-syn in absence or presence of 1.5 mg/ml of KO cytosol. As shown on this graph, A30P purified α-syn has a lower binding compared to Wt and A53T α-syn in absence (One-Way ANOVA, p < 0.0001, n = 4; Bonferroni's multiple comparison test) or presence (One-Way ANOVA, p < 0.0001, n = 4; Bonferroni's multiple comparison test) of KO cytosol. **(C) **KO synaptic membranes were incubated, for 10 min at 37°C, with 0.1, 0.6 and 3 μg of Wt, A30P or A53T purified α-syn in absence or presence of 1.5 mg/ml of KO cytosol. Results are normalized to the maximal binding observed for each respective α-syn. These data show that the cytosol has a significant effect by increasing the binding of all types of α-syn (One-Way ANOVA: Wt: p < 0.0001, n = 4; A30P: p < 0.0001, n = 4; A53T p < 0.001, n = 4).

## Methods

### Synaptosome preparation

Synaptosomes were prepared as described (Fischer von Mollard et al. 1991;Tandon et al. 1998a). Briefly, the cerebral cortices from mice α-syn KO mice were dissected and homogenized with 10 strokes at 500 rpm, in ice-cold buffer A (320 mM sucrose, 1 mM EGTA, and 5 mM HEPES [pH 7.4]). The homogenate was centrifuged at 1000 × g for 10 min. Next, the supernatant was spun for 10 min at 24000 × g and the resulting pellet (P2) resuspended in buffer A. The P2 fraction was loaded onto a discontinuous FICOLL gradient (13%, 9%, 5% in buffer A) and centrifuged for 35 min at 35,000 × g. The 13%-9% interface, containing intact synaptosomes, was resuspended in buffer B (140 mM NaCl, 5 mM KCl, 20 mM HEPES, 5 mM NaHCO3, 1.2 mM Na2HPO4, 1 mM MgCl2, 1 mM EGTA, and 10 mM glucose). The sample was spun at 24000 × g for 10 min and the pellet was washed two times in buffer C (10 mM HEPES, 18 mM KOAc, [pH 7.2]), then spun at 24000 × g for 10 min and resuspended in buffer D (25 mM HEPES, 125 mM KoAc and 2.5 mM MgCl_2_). After centrifugation (24000 × g for 10 min), synaptosomes were resuspended in buffer D and were incubated with or without brain α-syn KO cytosol. Samples were incubated for 10 min at 37°C before separating membrane and supernatant by centrifugation at 24000 × g for 10 min. α-syn binding was quantified by western blotting.

### Cytosol preparation

Mouse brains were thoroughly homogenized in 85 mM sucrose, 100 mM KOAc, 1 mM MgOAc, and 20 mM HEPES (pH 7.4). The homogenate was centrifuged for 10 min at 15,000 × g and the supernatant spun for 1 hr at 100,000 × g. The supernatant was subsequently dialyzed for 4 hr in 145 mM KOAc and 25 mM HEPES (pH 7.2) and frozen at -80°C. Protein concentration was determined by BCA protein assay (Pierce, Biolynx Inc., Canada).

### Lipid-free cytosol preparation

Chloroform was added to the cytosol (v/v), vigorously vortexed and incubated for 30 min at room temperature. After centrifugation for 10 min at 14000 × g, two phases were obtained: upper phase (TOP) containing the gangliosides or small organic molecules, the interphase containing the proteins and the lower phase containing the lipids. In some experiments, 1-O-hexadecyl-2-acetyl-*sn*-glycero-3-phosphocholine (C16:0 PAF, Biomol) was added alone or directly to delipidated cytosol to test effect on α-syn membrane binding.

### Cytosol digestion

Cytosol digestion was done with trypsin or Proteinase K and proteolytic activity was terminated with trypsin inhibitor or PMSF, respectively prior to the incubation with membranes. The enzyme inhibition was controlled by a partial rescue of the digested cytosol after half-dilution with untreated cytosol.

### Expression and Purification of Recombinant α-synuclein

Human Wt α-syn cDNAs were subcloned into the plasmid pET-28a (Novagen), using Nco I and Hind III restriction sites. α-Syn was overexpressed in Escherichia coli BL21 (DE3) via an isopropyl-1-thio-3/4-D-galactopyranoside-inducible T7 promoter. The bacterial pellet was resuspended in phosphate buffered saline (PBS) containing 1 mM phenylmethylsulfonyl fluoride (PMSF). The bacterial suspension was then sonicated for 30 sec several times, boiled for 15 min, and ultracentrifuged at 150,000 × g for 30 min. The supernatant containing the heat-stable α-syn was dialyzed against 50 mM Tris, pH 8.3, loaded onto a Q-Sepharose column (Pharmacia Biotech), and eluted with a 0–500 mM NaCl step-gradient. The eluents were desalted and concentrated on a Centricon-10 (Millipore) in 5 mM phosphate buffer, pH 7.3. Aliquots of each purification step were analyzed by SDS-polyacrylamide gel electrophoresis (PAGE) to confirm purity. Protein concentration was determined by Lowry assay.

### Western blotting

Proteins were boiled briefly in loading buffer (glycerol 10% v/v; Tris 0.05 M pH 6.8; SDS 2%, bromophenol blue and 2.5% v/v β-mercaptoethanol) and separated by electrophoresis using 12% Tris-glycine polyacrylamide gels. Proteins were transferred to nitrocellulose (Life Sciences) and probed by western blotting using: antibodies against α-syn (monoclonals 211 and Syn-1 at 1:1000, Neomarkers), our own rabbit polyclonal (LWS1, 1:1000) raised to a 24-mer α-syn-specific peptide, or synaptophysin (Mouse monoclonal antibody, dilution 1:10000, Biodesign International). Bound HRP-conjugated anti-mouse or anti-rabbit IgG (Sigma) were revealed by chemiluminescence using ECL Plus (GE Healthcare) and quantified with a Storm 860 fluorescent imager and ImageQuant software (Molecular Dynamics). Statistical comparisons were calculated with GraphPad InStat software using Student's T-test for comparisons between two groups or ANOVA (Bonferroni test) for multiple comparisons.

### Synaptic lipid raft preparation

Lipid rafts were prepared from the synaptosomes or synaptic membrane isolated from cortices as described above. Synaptosomes or synaptic membrane were resuspended in 25 mM MES, pH 6.5, 50 mM NaCl, 1 mM NaF, 1 mM Na3VO4, and 1% TX-100 (lysis buffer) supplemented with phosphatase inhibitor cocktails (Sigma) and incubated on ice for 30 min with Dounce homogenization every 10 min. The cell lysate was then adjusted to 42.5% sucrose, overlayed with 35 and 5% sucrose in lysis buffer without TX-100 and sedimented at 275,000 × *g *for 18 hr at 4°C. Fractions were collected from the top of the gradient and stored at -80°C. Equal volumes of each fraction were separated by sodium dodecyl sulfate-polyacrylamide gel electrophoresis (SDS-PAGE) and probed with the different antibodies as described above. Lipid raft-containing fractions were identified by the presence of flotillin-1 (BD Biosciences, Canada).

### Glycerophospholipid extraction

C13:0 lysophosphatidylcholine (C13:0 LPC) and 1-*O*-hexadecyl-2-[^2^H_4_]acetyl-glycerophosphocholine (d_4_-16:0 PAF) were purchased from Avanti Polar Lipids (Alabaster, AL). Stock chemicals were purchased from J.T. Baker (Phillipsburg, NJ) with the exception of bovine serum albumin (BSA) from Sigma (St. Louis, MO). Glycerophospholipids were extracted according to a modified Bligh/Dyer procedure [15] as we have previously published[16]. Briefly, lipids were extracted using a volumetric ratio of 0.95 of chloroform and 0.8 of 0.1 M Na acetate (aq) per volume of MeOH in acid-washed borosilicate glass tubes (Fisher, Ottawa, ON). Phospholipids were collected from the organic phase after layer separation by centrifugation. The aqueous phase was back-extracted three times in the organic phase of a wash solution prepared by combining RPMI+ 0.025% BSA, methanol, chloroform, and sodium acetate in the volumetric ratio of 1:2.5:3.75:1. The organic fractions were combined, evaporated under a stream of nitrogen gas, and dissolved in 300 μl EtOH. C13:0 lysophosphatidylcholine (C13:0 LPC), a lipid not naturally occurring in mammalian cells [17], was spiked into cytosol preparations at a concentration of 189 ng prior to extraction to control for variation in extraction efficiency.

### LC-ESI-MS

Glycerophospholipids were analyzed as we have described previously [16]. Briefly, extracts were diluted 1:4 in EtOH with 13 μL of diluent brought to 40 μl with 0.1% formic acid in H_2_O. To validate the identity of target species, analytes were spiked with 1-*O*-hexadecyl-2-[^2^H_4_]acetyl-glycerophosphocholine (d_4_-16:0 PAF, 2.5 ng) in replicate LC-ESI-MS/MS analyses. Under these circumstances, 10 μl of diluted analyte was added to 5 μl of standard (2.5 ng) and brought to 40 μl with 0.1% formic acid in H_2_O. Samples were loaded onto a 96-well sampling plate, covered with a pre-slit well cap, and thermostated at 4°C. A micro flow 1100 HPLC system (Agilent, Palo Alto, CA) introduced the analytes onto a 200 um × 50 mm pre-column packed with 5 μm YMC ODS-A C18 beads (Waters, Milford, MA) at a flow rate of 10 μl/min in a 2000 Q TRAP mass spectrometer. The solvents used were water and acetonitrile each with 0.1% formic acid (J.T. Baker, Phillipsburg, NJ). The HPLC flow was split and the analyte was eluted through a 75 um × 50 mm picotip emitter (New Objective, Woburn, MA), interfaced with the mass spectrometer via electrospray ionization, at ~200 nL/min. The emitter was packed with the same beads as those of the pre-column. A linear gradient was used to separate glycerophospholipid species. The gradient of the HPLC increased from 5% to 30% acetonitrile in 2 minute, from 30 to 60% acetonitrile in 7 minute, from 60% to 80% acetonitrile over the next 33 minutes, and from 80% to 95% acetonitrile over the next 4 minutes. Data were collected on a 2000 Q-TRAP mass spectrometer operated with Analyst 1.4.1 (Applied Biosystems/MDS Sciex, Concord, ON). Total glycerophospholipids between m/z range of 450 to 600 were analyzed by enhanced MS scan. Specific glycerophosphocholine species were further analysed in positive ion mode using precursor ion scan for an MS/MS fragment with a mass to charge ratio (m/z) of 184.0, a diagnostic fragment of phosphocholine [18]. Extracted ion chromatogram (XIC) generated peak areas of LC-MS/MS data measured using Analyst 1.4.1 (Applied Biosystems/MDS Sciex). Peak areas were normalized to the spiked internal standard to standardize between MS runs and to control for variation in extraction efficiency. Individual species were identified based on theoretical mass validated by closer examination of retention time and following spiking with deuterated standards.

## Results

### Cytosol modulates α-syn membrane binding

To identify novel co-factors of α-syn binding to presynaptic membranes, we assessed whether co-incubation with brain cytosol modifies α-syn's interaction with membranes. Our assay measured the binding of recombinant human α-syn purified from E. coli to synaptic membranes prepared from brains of α-syn-deficient (KO) mice, in the presence or absence of brain cytosol derived from α-syn-deficient mice (Figure 1A). We first analysed α-syn binding to synaptic membranes in the presence or absence of cytosol. As shown in Figure 1B, the binding of α-syn, with or without familial PD-linked mutations, was significantly improved by co-incubation with cytosol. Despite the deficient membrane binding of A30P as compared to that of Wt and A53T, all three forms of α-syn showed increased binding over a 30-fold range in concentration, with a pronounced augmentation of binding in the presence of cytosol (Figure 1C). The ratio of bound/unbound α-syn was higher at lower α-syn concentrations. These results suggest that endogenous cytosolic factors becoming limiting with increasing α-syn and can partially counterbalance the otherwise impaired binding induced by the A30P mutation.

### Characterization of cytosol action on α-syn binding

We recently reported that the dissociation of the α-syn from synaptic membranes requires cytosolic proteins as defined by sensitivity to proteases. To further characterize cytosol action on α-syn binding, and because the data in Fig 1C suggests that cytosol activity becomes saturated at high α-syn concentration, we analysed α-syn binding with varying cytosol concentrations over a 6-fold range that we have previously shown to be effective in mobilizing reserve neurotransmitter from permeabilized synaptosomes [19] (Figure 2A). In accord with the data in figure 1B, both Wt and A30P α-syn binding was strongly up-regulated by increasing cytosol concentration, whereas only high cytosol concentration resulted in increased A53T α-syn binding. To determine whether the cytosolic factors act on α-syn or on the acceptor synaptic membranes, we first pre-incubated α-syn or synaptic membranes separately with KO cytosol. The membranes were subsequently washed briefly to remove unbound cytosolic factors. As shown on Figure 2B, exposure of the membranes alone to cytosol was sufficient to potentiate α-syn binding, which was equivalent to α-syn binding to membranes in the presence of cytosol. These results suggest that cytosolic activity can be mediated by affecting the acceptor membrane rather than soluble α-syn.

**Figure 2:** **Effect of cytosol on binding α-syn**. **(A) **Recombinant α-syn (Wt, A30P and A53T) were incubated in presence of different concentrations of KO cytosol (0.5, 1.5, and 3 mg/ml), for 10 min at 37°C. Compared to the control condition (without cytosol), all cytosol concentrations had a significant effect on Wt and A30P α-syn binding, but only the highest concentration of cytosol had a significant effect on A53T α-syn binding (One way ANOVA test, p < 0.0001, Bonferroni's multiple comparison post-test). **(B) **KO synaptic membranes and α-syn were pre-incubated for 15 minutes at room temperature with KO cytosol. Membranes were then centrifuged at 14000 × g and washed with KOAc buffer to remove unbound factors. Binding of purified α-syn to KO membranes in the absence of cytosol (ctrl) was compared to its binding to cytosol-treated membranes without added cytosol (memb), and to cytosol-treated α-syn incubated with KO membranes (α-syn). No significant difference was observed between the two pre-incubated condition (Student T-test, p > 0.05). **(C) **KO cytosol was pre-incubated with trypsin or proteinase K for 15 min at 37°C. Enzymes were then respectively inactivated with trypsin inhibitor and PMSF for 10 min at room temperature. Compared to the cytosol condition (cyt) which, as a control, was incubated with the enzyme pre-inactivated by the inhibitor, only A30P α-syn binding was significantly affected by the cytosolic protein digestion (Student T-test, p < 0.0001), whereas no significant differences were observed for Wt and A53T proteins (Student T-test, p > 0.05).

To determine the nature of the cytosolic factor(s), we assessed whether activity was affected by pre-digestion of cytosolic proteins by trypsin- or proteinase K-mediated proteolysis (Figure 2C). Digestion of cytosol was terminated by trypsin inhibitor and PMSF prior to incubation with α-syn and synaptic membranes, and the extent of proteolysis was verified by Coomassie blue stain (not shown). Although, no significant differences between undigested and digested cytosol were observed for either Wt or A53T α-syn binding, the A30P mutant showed significantly reduced binding in the presence of protease-treated cytosol, reaching a basal level similar to the control condition in absence of cytosol. This suggests that the A30P mutation confers a unique dependence on cytosolic protein(s) required to mediate α-syn interactions with synaptic membranes. Moreover, comparable levels of a non-specific protein, bovine serum albumin (BSA), did not affect A30P α-syn binding to synaptic membranes (data not shown), suggesting that A30P α-syn binding depends on specific cytosolic proteins.

### Involvement of cytosolic lipids in α-syn membrane binding

Because Wt and A53T α-syn appear to require protease-insensitive cofactors for membrane binding, and α-syn conformation is known to be affected by lipids (Jo et al. 2002), we examined whether removal of cytosolic lipids by chloroform extraction can alter the proportion of α-syn able to bind synaptic membranes (Figure 3A). We observed that the binding of Wt α-syn and PD-linked mutants were decreased in the presence lipid-deficient cytosol, suggesting a role for cytosolic lipids in the binding of α-syn to synaptic membranes. These results are also consistent with our observation that heat-denatured cytosol retains its activity to potentiate Wt and A53T α-syn binding (data not shown). Moreover, consistent with the results in Fig 1B showing that A53T α-syn membrane binding is less dependent on cytosol, it was also the least affected by lipid extraction. It is also important to note that the chloroform extraction did not non-specifically denature cytosolic proteins because the protein-containing fraction partially rescued A30P α-syn binding, in accord with its dependence on a protease-sensitive cytosolic component.

**Figure 3:** **Effects of cytosolic lipid depletion on α-syn binding**. **(A) **Using chloroform extraction to fractionate cytosol into three fractions: the top fraction contains the gangliosides or small organic polar molecules, the interface layer contains the proteins and the bottom phase contains lipids solubilised in chloroform. We incubated the synaptic membrane with the two lipid free-fractions, top and interphase (protein) layers, in presence of recombinant α-syn. The lipid-free fractions did not show any significant effects on the Wt and A53T α-syn binding compared to the control condition (α-syn incubated with synaptic membranes in absence of cytosol; Student T-test, p > 0.05) while the A30P α-syn binding was increased (compared to control condition, Student T-test, p < 0.01). **(B) **Recombinant α-syn (Wt, A30P and A53T) were incubated with synaptosomal membranes in the presence of 1.5 mg/ml cytosol from either KO mice (KO) or from non-transgenic mice (nonTg) for 10 min at 37°C. Binding of normal and mutant human α-syn, measured by the human α-syn specific monoclonal antibody 211, is normalized to that of Wt α-syn in the presence of KO cytosol. **(C) **Recombinant Wt α-syn was incubated with synaptosomal membranes and C16:0 PAF (0, 10, 100 nM) in the absence (open bars) or presence of delipidated cytosol (closed bars). Inclusion of 100 nM C16:0 PAF significantly increased α-syn binding only in the presence of the delipidated cytosol (compared to corresponding condition without C16:0 PAF, Two-Way ANOVA, p < 0.01, Bonferroni's multiple comparison test p < 0.01, n = 3).

Several studies have noted significant changes in brain lipids, notably in the metabolism of neutral brain lipids, in α-syn-deficient animals [20-22]. Therefore, to test whether our results are specific to KO cytosol we compared human α-syn binding in the presence of KO cytosol or cytosol derived from nontransgenic animals with normal α-syn expression. In order to detect only the exogenously added human α-syn, and not endogenous murine α-syn present in normal cytosol, we used the human α-syn specific monoclonal antibody 211. We observed no significant differences in cytosol-dependent α-syn binding when KO versus normal cytosol was used (Figure 3B).

We used LC-ESI-MS to identify lipid cofactors present in α-syn KO cytosol. Because previous studies have indicated that the strongest lipid interactions with α-syn are with either neutral or anionic phospholipids [3,8,23,24], we focused our initial analysis on the glycerophosphocholine species present in KO cytosolic extracts [18] as the detection methodologies are well-established in our laboratory [16]. As our extracts are dialyzed prior to testing, these lipid species are predicted to be in complexes with proteins greater than 12 kDa. Choline-containing lipids extracted from these complexes were separated and species with a mass to charge ratio (m/z) between 450 and 600 identified by MS scan for a protonated molecule at expected m/z followed by positive ion mode precursor ion scan for a phosphocholine product ion at m/z 184 [16]. Twenty-four candidate species were identified in the extracted ion chromatographs (Table 1). Because α-syn is known to play a role in regulating lipid metabolism in brain, notably in the regulation of the glycerophosphocholine fatty acid turn over, [21,22,25,26], we compared this profile to the lipids detected in Wt cytosol. We found that Wt cytosol contained the same glycerophosphocholines as KO preparations with the exception of two species detected *de novo *(Table 1). The overall abundance of the majority of small second messenger species was elevated in KO cytosol relative to Wt.

**Table 1:** Elution time and parent ion masses of candidate glycerophosphocholine species bound to proteins in dialyzed α-synuclein KO cytosolic extracts identified by LC-ESI-MS

*Parent ion mass (± 0.15 m/z)^a^*	*LC elution time (± 0.4 min)^a^*	*Lipid species in complex with proteins in KO cytosol^b^*	*Species abundance relative to Wt (Fold change)*	*Species bound to α-syn following immunoprecipitation (Fold change above non-specific binding)^c^*
494.7	12.29	C14:1-PAF	↑-fold	
	12.89	C16:1-LPC	No change	
496.8	13.79	C14:0-PAF	↑3-fold	↑9.2^x^
	14.39	C16:0 LPC	↑2-fold	↑9.8^y^
520.7	13	C16:2-PAF	↑2-fold	
	13.41	C18:2-LPC	No change	
522.8	14.66	C16:1-PAF	↑5-fold	
	15.15	C18:1-LPC	↑2-fold	
524.9	17.2	C16:0-PAF^c^	↑2-fold	↑1.7x
	18.11	C18:0-LPC	↑4-fold	↑2.3y
545		C18:4-PAF	↑11-fold	
	13.12	C20:4-LPC		
545.9	13.11	C18:3-PAF	*De novo detection*	
	13.99	C20:3-LPC		
568.8	13.12	C20:6-PAF	↑4-fold	
		C22:6-LPC		
581	15.32	C20:0-PAF	↑17-fold	
	16.04	C22:0-LPC	↑12-fold	
594	16.52	C24:7-LPC	↑2-fold	
		C22:7-PAF		
		23:7c		
		24:7d		
		C20:0-acyl-PAF		
		C24:0-lysoPAF		

^***a ***^Variations between *m*/*z *and retention time between runs were established for all glycerophospholipid species and respresents mean ± standard deviation.

^***b ***^Identification is predicted based on the theoretical monoisotopic mass values. C*X*:*Y *refers to the number of carbon atoms and double bonds in the *sn*-1 chain with a predicted acetyl (PAF) or hydroxyl (LPC) group at the *sn*-2 position. Only the most likely species are indicated although multiple isoforms may be present with the double bond in the alkyl chain at different positions. Isobaric species with same m/z eluting at different times were not further distinguished with the exception of C16:0 PAF.

^***c ***^Replicate experiments were performed in which α-syn was immunoprecipitated from Wt cytosol^*x *^or recombinant α-syn was added to KO cytosol^*y*^. Immunoprecipitates were analysed by LC-ESI-MS. Data represent mean increase in relative abundance above background (non-specific) signal ± standard deviation as described in Materials and Methods.

^***d ***^Identity verified by based on its coelution with d_4_-C_16_-PAF spiked at time of analysis.

To identify glycerophosphocholines interacting directly with α-syn in our binding assays, we performed two complementary analyses. First, we immunoprecipitated α-syn from Wt cytosol and identified the glycerophosphocholine present in protein complex after dialysis by LC-ESI-MS. Second, we incubated recombinant α-syn with KO cytosol and identified lipid binding partners following immunoprecipitation. Non-specific lipid binding was assessed by lipid analysis of immunoprecipitates for α-syn from KO cytosol. Data are expressed as fold change in lipid abundance above background (Table 1). Only two predicated species exhibited significant association with Wt and Wt recombinant α-syn: C14:0 PAF and C16:0 PAF. C16:0 PAF was definitively identified by based on its co-elution with d_4_-C_16_-PAF (m/z 528.7) (data not shown). C14:0 PAF was identified based on retention time and monoisotopic mass values. Definitive identification was not possible in the absence of a commercially available synthetic standard of suitable purity. To validate effects of C16:0 PAF on α-syn membrane interaction, we tested whether C16:0 PAF enhanced α-syn binding to synaptic membranes directly (Fig 3C). Incubation of α-syn with C16:0 PAF alone did not affect α-syn membrane binding. However, when C16:0 PAF was added in combination with delipidated cytosol, α-syn binding was significantly increased. This data are suggestive of a protein-lipid complex required to enhance α-syn's capacity to interact with neuronal membranes. Specificity was tested using C16:0 *lyso*-PAF that differs from PAF by the presence of an hydroxyl group in place of an acetyl group at the *sn*-2 position. C16:0 *lyso*-PAF was not detected by LC-ESI-MS analysis in complex with protein in KO cytosol or α-syn immunoprecipitates and did not enhance α-syn membrane binding alone or in combination with delipidated cytosol (data not shown).

### A30P Parkinson's disease-linked mutation interacts differently with synaptic membranes compared to Wt

Our results above, though consistent with previous reports showing that the A30P mutation impairs membrane binding ability compared to Wt and A53T α-syn, notably indicate that A30P α-syn binding is also significantly enhanced by cytosol, albeit not to the extent of Wt α-syn. Because α-syn is prone to self-aggregation and changes to the secondary structure of α-syn could induce artifactual differences between Wt, A53T and A30P membrane binding, we assessed whether each of the α-syn proteins are structurally similar in their soluble form prior to exposure to membranes, and not dimerized or aggregated which could affect membrane binding ability. All three α-syn proteins eluted in the same fractions as monomers from a size-exclusion column, and their circular dichroism spectra showed the characteristic minima of a randomly structured protein near 200 nm (Figure 4).

**Figure 4:** **Purified E-coli α-syn is monomeric and unstructured**. Each recombinant α-syn (Wt, A30P and A53T) was analyzed by size exclusion chromatography to determine the presence of monomeric, dimeric, or other higher order forms. Eluate peaks (fraction 27) were then assessed by circular dichroism spectra to define the secondary structure of the α-syn proteins (Inset). Far-UV circular dichroism spectra were recorded on an Aviv circular dichroism spectrometer model 62DS (Lakewood, NJ, USA) at 25°C using quartz cells with a path length of 0.1 cm. Spectra were obtained from 195 nm to 260 nm, with a 1.0-nm step, 1.0-nm bandwidth, and 4-s collection time per step. The experimental data were expressed as mean residue ellipticity (θ) (deg·cm^2^·dmol^-1^). Only monomeric forms of α-syn where identified by size exclusion chromatography, and all α-syn share similar random secondary structure.

Previous *in vitro *studies using artificial or cellular membranes showed that α-syn interacts with lipids and preferentially associates with lipid raft fractions isolated from cultured HeLa cells or synaptic vesicles [27,28]. Moreover, in those studies the A30P mutation impaired interaction with rafts, and consequently, with the membrane. Because those studies evaluating α-syn membrane binding did not assess cytosolic co-factors that could ostensibly regulate α-syn behaviour *in vivo*, we analysed the proportion of purified α-syn recovered with the lipid raft fractions following binding in the presence or absence of KO cytosol (Figure 5A). In contrast to the previous report [28], we found that very little exogenously-added α-syn (< 5%) co-eluted with the flotillin-positive lipid raft fractions, and this was not affected by the presence of cytosol, although α-syn immunoreactivity in other fractions (6–9) was increased by cytosol. These results indicate that the cytosol-dependent change in α-syn membrane binding was not due to increased association with lipid rafts, and the A30P α-syn was not less likely to co-elute with flotillin-rich fraction than either Wt or A53T α-syn.

**Figure 5:** **α-Syn binding to synaptosomal lipid rafts**. Using a 42-30-5% discontinuous sucrose gradient, we analysed the proportion of α-syn that co-localised with flotilin-1, a lipid-raft marker. **(A) **Less then 5% of α-syn co-eluted with flotillin-1 after binding (*in vitro*) to α-syn KO synaptic membranes, in absence or presence of KO cytosol, and proportionally, no significant differences were observed between Wt and PD-linked mutants (Student's T-test, p > 0.05). **(B) **The proportion of α-syn that co-localised with flotillin-1 *in vivo*, using intact synaptosomes from transgenic mice expressing the human α-syn (Wt, A30P or A53T). As observed *in vitro*, only a small proportion of α-syn co-eluted with lipid rafts and no significant differences were observed between Wt and PD-linked mutations (Student T-test, p > 0.05). **(C) **A30P α-syn was subjected to paraformaldehyde-induced cross-linking to potential interacting proteins in synaptic membranes after 1, 2, 3, 5 and 10 minutes of incubation with synaptic membranes. A significant increase of bound α-syn after 2, 3 and 5 minutes was observed compared to the control condition (without cross-linking) (One-Way ANOVA p < 0.001, Bonferroni's multiple comparison test). **(D) **The proportion of α-syn present in the lipid-raft fraction after cross-linking did not show any significant differences compared to incubations without cross-linking (Student t-test: 1 min: p > 0.05; 3 min: p > 0.05). **(E) **A significant increase of bound Wt and A53T α-syn after paraformaldehyde-induced cross-linking was observed compared to the control condition without cross-linking (One-Way ANOVA, *p < 0.05, **p < 0.01,***p < 0.001, Bonferroni's multiple comparison test).

To assess whether endogenously expressed cytosolic factors might play a role in regulating α-syn association to lipid rafts *in vivo*, but are not fully reproduced in our *in vitro *assay, we also quantified the amount of α-syn that co-elutes with flotillin-1 in synaptosomes from brains of human α-syn Tg mice. Only a minor fraction of total α-syn co-eluted with the lipid raft fraction from mouse brain synaptosomes (Figure 5B) or from whole brains (not shown), and we observed no significant differences between both PD mutants and Wt α-syn. Thus, mouse brain-expressed A30P α-syn appears to show a similarly weak distribution (< 5%) to gradient fractions containing lipid raft marker flotillin-1 as Wt and A53T α-syn.

We also considered the possibility that the lower binding of A30P α-syn to total membranes is due to a transient or low affinity interaction that is not stable during isolation. To test this hypothesis, we assessed whether covalent cross-linking using paraformaldehyde after different incubation periods with purified A30P α-syn might stabilize the bound α-syn. Under these conditions, cross-linking increased α-syn association at t = 2, 3 and 5 minutes (Figure 5C). This additional α-syn was mostly excluded from the gradient fractions containing lipid rafts (Figure 5D) suggesting that the α-syn binding to membranes may be stabilized by other membrane proteins but not those associated with lipid rafts. Similar to the A30P mutant, Wt and A53T α-syn binding to membrane was also increased by cross-linking (Fig 5E). However, maximal binding of the Wt α-syn occurred in the first minute and remained stable thereafter. The binding of A53T mutant also peaked in first minute, but then slowly declined. Thus, the binding kinetics of α-syn bearing either PD-linked mutation suggest a more transient membrane interaction.

### α-Syn interaction with synaptic membrane is regulated by ATP

α-Syn membrane attachment may be regulated by nerve terminal activity initiated by membrane depolarization [27], a process which results in Ca^2+ ^influx, and elevated metabolic energy consumption. Therefore, we tested whether the addition of Ca^2+ ^and ATP influenced α-syn binding. Our results show that ATP, but not ATPγS, significantly increased the level of membrane bound Wt α-syn and PD-linked mutants in the absence or presence of KO cytosol, whereas Ca^2+ ^had no affect the α-syn binding (Figure 6A–C). The effect of ATP was additive to cytosol action suggesting that they act independently, and this was supported by the fact that ATPγS did not reduce the cytosol-dependent binding.

**Figure 6:** **(A-C) **Recombinant α-syn (Wt, A30P and A53T) were incubated with ATP (1 mM), ATPγS (3 mM), Ca^2+ ^(1 mM), ATP/Ca^2+ ^or ATPγS/Ca^2+ ^in absence or presence of 1.5 mg/ml of KO cytosol, for 10 min at 37°C. Incubation with ATP (Student's T-test, p < 0.001), but not ATPγS or Ca^++ ^(Student's T-test, p > 0.05), induced a significant increase in the binding of Wt and mutant forms of α-syn (compared to control condition without added cofactors).

## Discussion

Aberrant aggregation of α-syn has been detected in an increasing number of neurodegenerative diseases, now collectively known as synucleinopathies. These include Parkinson's disease (PD), Dementia with Lewy bodies (DLB), Alzheimer's disease (AD), multiple system atrophy, and Down syndrome [29]. Accumulations of α-syn in all these disorders have a common fibrillar configuration, though they differ in the co-localisation with other proteins including tau, parkin, and synphilin [30]. While the physiological functions of normal α-syn remain to be fully elucidated, several studies suggested it may play a role in synaptic plasticity, regulate dopamine (DA) neurotransmission via effects on vesicular DA storage, and act as a co-chaperone with cysteine-string protein to maintain nerve terminals [31]. These roles may involve α-syn interactions with proteins in cytosol and on membranes, though little is known about the α-syn membrane interaction *in vivo *and how membrane-bound and freely-diffusible pools of α-syn are maintained. Therefore, to understand the regulation of α-syn interaction with synaptic membranes, we developed an *in vitro *assay which measures the binding of recombinant *E. coli*-derived α-syn to α-syn-deficient synaptosomal membranes and recapitulates many features of the interactions observed *in vivo*.

Using this binding assay, we showed that approximately 60% of the Wt and A53T soluble α-syn interacts with membrane, whereas only a small amount of the PD-linked A30P mutant is able to stably bind to the membrane (Figure 1B). Reduced A30P binding has been well-reported in several studies using artificial membranes [32-34] and can be explained by the expected disruption of the α-helix induced by the mutation. Indeed, the secondary structure of α-syn is divided into an α-helical lipid-binding amino-terminal and an unstructured lipid-free carboxyl-terminal [35]. The replacement of an Ala by a Pro in the A30P variant restricts the conformational space available to the preceding residue, Ala29, implying the loss of two intra-helical hydrogen bonds modifying the backbone structure of the protein, while the backbone structure and dynamics of the A53T α-syn mutant is found to be virtually unchanged from the Wt [36].

Despite the predicted structural limitations induced by the A30P mutation, and its impaired membrane binding capacity noted in *in vitro *assays, we showed previously that the amounts of Wt, A53T, and A30P α-syn that segregate with synaptic membrane fractions derived from mouse brains are not significantly different [14]. These disparate findings suggest that additional factors *in vivo *control α-syn membrane binding and can be reconciled by our present results showing that the addition of mouse brain cytosol stimulated the membrane association of Wt and A53T α-syn and partially rescued the intrinsically poor binding of the A30P α-syn. These data provide evidence that the subcellular proportion of membrane-bound and soluble α-syn may be regulated by cytosolic factors *in vivo*, which are far more concentrated (~300 mg/ml) than the 0.5–3 mg/ml cytosol used in our assay, and might compensate for the low A30P α-syn membrane association observed *in vitro*.

Surprisingly, we observed that pre-exposure of membranes to cytosol was sufficient to augment subsequent α-syn binding, suggesting a mechanism whereby membranes can be primed by cytosolic factors for α-syn recruitment. Moreover, unlike the cytosolic protein requirement for the dissociation of α-syn from synaptic membrane [14], the cytosol-dependent component of α-syn binding is resistant to digestion by proteinase K and trypsin for the Wt and A53T α-syn, though not for A30P α-syn. This suggests that although cytosolic proteins are not required for the Wt and A53T α-syn membrane interaction, α-syn with A30P mutation would require protein assistance. As it is unlikely that a specific protein interaction evolved to specifically maintain A30P α-syn binding, the protein interaction implied by our results may also interact with Wt α-syn as well, though it is not essential for its membrane binding. We previously reported that cytosolic proteins are required for the dissociation of membrane-bound α-syn [14], presumably by transient association with α-helical conformation of α-syn on lipid bilayers. The same factor(s) may also aid in the reverse reaction by coordinating the A30P α-syn amino terminal to configure into an amphipathic α-helix so as to overcome its conformational limitations or to stabilize the mutant in closer apposition to the lipid bilayer prior to membrane binding. Such a mechanism could also account for the transient interaction we observed for A30P mutant with the membrane fraction. By briefly inducing covalent cross-links at various times to stabilize bound α-syn, we observed that A30P α-syn binding was biphasic, peaking at 3 min and declining thereafter. It is important to note this was not due to non-specific cross-linking because the later incubation periods (i.e. 10 min) did not show increased recovery of A30P α-syn with membranes despite the substantial soluble A30P α-syn. These results suggest that α-syn membrane binding may be partially coordinated by local synaptic vesicle proteins. Indeed, proteins such as cysteine string protein or members of the Rab family may fulfil this role [31,37,38]. Cross-linking also increased the recovery of bound Wt and A53T α-syn, although the kinetics were different from the A30P mutant. Both Wt and A53T binding peaked in the first minute of incubation suggesting a quicker interaction with synaptic membranes. Interestingly, the Wt α-syn remained stably associated even when cross-linking was activated after 10 min of incubation, the A53T binding declined slowly. These results are consistent with our previous report [14] showing greater cytosol-dependent dissociation of both PD mutants from synaptic membranes.

In the course of characterizing the protein-dependence, we noted that lipid-depleted cytosol lost its activity to induce α-syn binding. Because the cytosol used in these experiments is dialyzed using membranes with a 12 kDa molecular weight cut-off, only lipid-protein complexes larger than 12 kDa are retained. These results suggested that protein-bound polar lipids are likely the protease-insensitive cytosolic components responsible for assisting the membrane binding of α-syn. In accord with the conformational model of α-syn [39,40] whereby it acquires a folded helical structure in the N-terminal region in its membrane-bound state, our results suggested that endogenous cytosolic lipids transferred to membranes prior to α-syn recruitment or bound directly to cytosolic α-syn may aid α-syn folding at the lipid-cytoplasm interface so it is more amenable to binding directly to synaptic membranes. To provide further insight into this novel protein-lipid-protein interaction, we profiled glycerophosphocholines bound to proteins in α-syn-deficient cytosol by nanoflow LC-ESI-MS and precursor ion scan. Our analysis identified 24 species that can potentially affect α-syn membrane interactions. While this number clearly underestimates the cytosolic lipid content *in vivo *given our MS analyses were limited to polar glycerophospholipids with an m/z between 450 and 600, of which glycerophosphocholine-containing species were further analyzed, these data represent the first profile of candidate lipid interactors at the molecular level responsible for the enhanced α-syn binding. Further, we demonstrated that two glycerophosphocholines C14:0 PAF and C16:0 PAF interact with α-syn, with C16:0 PAF definitively identified at the molecular level. Importantly, C16:0 PAF was able to rescue the ability of delipidated cytosol to potentiate α-syn membrane binding but did not, in and of itself, enhance α-syn interaction with membranes. This result suggests the involvement of a cytoplasmic protein, and although appears inconsistent with data in Fig. 2C showing that α-syn binding does not require intact cytosolic proteins, a more likely possibility is that a cytoplasmic protein may be required to activate or modify the exogenously added lipid. For example, binding to GM2 activator protein elicits a conformational change in PAF [41]. Arguably, endogenous PAF in brain cytosol would be active prior to the cytosol depletion, and thus delipidation, but not protein depletion, would impact a-syn binding. Similarly, addition of exogenous PAF, presumably in an inactive conformation, would need prior activation by delipidated cytosol. These findings are also consistent with previous studies indicating that α-syn does not directly bind to palmitic acid (C16:0) [25], yet addition of 1,2-palmitoyloleoylphosphatidylcholine to α-syn containing protein lysates promotes self-association and formation of protein complexes [24]. Here, we further confirmed specificity of these interactions using C16:0 *lyso*-PAF. C16:0 *lyso*-PAF did not impact α-syn interaction with neuronal membranes. Clearly, the nature of these protein-protein-lipid complexes and their effects on α-syn binding to synaptic membranes will require further investigation and expansion of the analysis of lipid co-factors beyond the small second messenger neutral glycerophosphocholines tested in this study. Careful analysis of these lipids will also be relevant to aging and neurodegeneration because abundant data suggest that cumulative oxidative modification of biomolecules, including lipids, plays an important role in aging, and free radical damage to brain lipids is involved in neuronal death in neurodegenerative disorders [42]. There is also accumulating evidence that α-syn deficiency has complex effects on brain lipid metabolism and production of lipid second messengers although the underlying mechanisms are poorly understood [20,21,25]. Consistent with these data, we also detected differences in PAF and LPC glycerophosphocholine levels between KO and normal cytosols, but these did not impact α-syn binding in our assay. Altogether, our data suggest that brain-lipids regulate α-syn binding, and an imbalance in specific species could mediate α-syn accumulation in the cytosol leading to fibril formation.

Despite previous studies suggesting that α-syn preferentially binds to lipid rafts in HeLa cells and to purified lipid raft fractions from rodent brain [27,28], we were unable to corroborate this interaction in our studies. We found that < 5% of total exogenously added α-syn co-eluted with the lipid raft marker flotillin-1, and this was unaffected by PD-linked mutations. Moreover, the same minor proportion of brain-expressed α-syn co-eluted with the flotillin-1 enriched fractions isolated from synaptosomes or whole brain, ostensibly reflecting negligible lipid raft associated α-syn *in vivo*. This low level of brain α-syn in lipid rafts was also noted by Fortin et al. [27], though they postulated that α-syn may dissociate from brain lipid rafts during the biochemical isolation. However, this explanation is inconsistent with the high recovery of overexpressed α-syn in lipid rafts from HeLa cells following the identical isolation procedure [27], and with our results showing that chemical cross-linking of A30P α-syn stabilized its membrane association, though not to lipid raft fractions. Two other explanations could account for the difference in the earlier studies and ours: First, lipid rafts in HeLa cells likely have a distinct lipid and protein composition compared to those in mammalian nerve terminals, possibly allowing them to bind overexpressed α-syn, which is not normally expressed in HeLa cells. Second, in the present work, lipid raft fractions were isolated only after α-syn was incubated with permeabilized synaptosomes, which retain sufficient internal architecture as to permit Ca^2+^-dependent exocytosis [19,43,44]. In contrast, the study by Kubo et al. [28] isolated lipid rafts before incubating with exogenous α-syn. The biochemical purification with 1% TX-100 likely modifies lipid rafts by altering lipid packing and/or loss of peripherally attached constituents, conceivably affecting subsequent α-syn binding capacity that is not normally present *in vivo*.

Because calcium influx and metabolic energy are both critical for the normal function of nerve terminals, we examined whether α-syn binding can be affected by modulating the availability of either Ca^2+ ^or ATP. We observed that α-syn binding has an ATP-dependant component that was not supported by ATPγS, and is insensitive to calcium. Because the increased α-syn binding in the presence of ATP and cytosol were additive and ATPγS did not affect cytosol-induced α-syn binding, it is likely that ATP and cytosolic factors act independently. One possibility is that ATP acts on a membrane protein whose interaction with membrane-bound α-syn is stabilized by chemical cross-linking, whereas cytosolic lipids modulate α-syn conformation either by direct interaction in cytosol or after intermediate transfer to a membrane component. Our results suggest that changes in synaptic ATP levels due to elevated metabolic consumption during exocytosis could modulate the α-syn solubility and may explain how neuronal depolarization can increase the level of freely-diffusible cytoplasmic α-syn in a Ca^2+^-independent manner [45]. The ATP sensitivity is also relevant to aging because neurodegenerative diseases are commonly associated with mitochondrial dysregulation and consequent impairment of energy production[46]. Under such pathological conditions, it is possible that lowered ATP levels may increase the cytosolic α-syn, which is significantly less constrained structurally than the membrane bound form. Concomitant oxidative stress could thereby promote β-sheet formation and accelerate α-syn aggregation.

## Conclusion

In conclusion, while the identities of the cytosolic components that assist the membrane interaction of α-syn remain to be fully characterized, our study reveals that cytosolic lipids and ATP are two of the principal factors regulating α-syn interaction with synaptic membranes. In addition, the relatively poor membrane binding of A30P α-syn could be explained by a more transient interaction with synaptic membrane and was partially rescued by the presence of protease-sensitive factors in brain cytosol. Those results suggest that endogenous brain proteins moderate the otherwise inefficient membrane association of A30P α-syn mutant, and represent a potential targets to influence α-syn solubility in brain.

## Abbreviations

α-syn: Alpha-synuclein; ESI-MS: electrospray ionization mass spectrometry; XIC: Extracted ion chromatogram; HPLC: High performance liquid chromatography; PD: Parkinson's disease; PAF: Platelet activating factor; Tg: Transgenic; Wt: Wild type.

## Authors' contributions

SW-G conducted the majority of the binding assays and drafted the manuscript; NPV contributed to the cross-linking and cytosolic lipid activity assays; SNW characterized the cytosolic and alpha-synuclein bound lipids; DM contributed to the alpha-synuclein purification and binding assays; WH and DF provided the MS data; PEF contributed reagents and participated in the circular dichroism analyses; SALB and AT designed and coordinated the study. All authors read and approved the final manuscript.
